The article "Based on Optimization Research on the Evaluation System of English Teaching Quality Based on GA-BPNN Algorithm" was published in 2022. Journal: Comput Intell Neurosci.

# Based on Optimization Research on the Evaluation System of English Teaching Quality Based on GA-BPNN Algorithm

**DOI:** 10.1155/2022/9946128

**Published:** 2022-01-05

**Authors:** Yafei Chen, Zhenbang Yu, Weihong Zhao

**Affiliations:** Qingdao Huanghai University, Qingdao, Shandong 266555, China

## Abstract

English teaching is an important part of basic teaching in our country, which has been deeply concerned by all aspects. Its teaching quality not only is related to the purpose of English teaching, but also has a far-reaching impact on students' English learning. Therefore, the construction of English teaching quality evaluation system has become the focus of research. However, the traditional English teaching quality evaluation method has some problems; for example, the subjectivity of teaching evaluation is strong, the evaluation index is not comprehensive, and the evaluation results are distorted. Therefore, this paper studies the English teaching quality evaluation system based on optimized GA-BP neural network algorithm. On the basis of BP neural network algorithm evaluation simulation, GA algorithm is introduced for optimizing, and GA-BP neural network algorithm model is further optimized by GA adaptive degree variation and entropy method. The experimental results show that the optimized GA-BP neural network algorithm has faster convergence speed and smaller error. At the same time, the optimized GA-BP neural network algorithm evaluation model has better adaptability and stability, and its expected results are more in line with the ideal value. The results of English teaching quality evaluation are more scientific, showing higher value in the application of English teaching quality evaluation.

## 1. Introduction

With the improvement of China's comprehensive strength, more and more people will choose to travel, work, and study, and more and more overseas people are willing to come to China for development. This not only promotes the economic exchanges between countries, but also makes the cultures of different countries constantly collide and exchange. Therefore, English teaching has been concerned by all walks of life. At present, English teaching in China has become one of the contents of basic education. There are different degrees of English teaching courses from primary school to university. Therefore, the quality of English teaching not only is related to the development of education, but also has a long-term impact on students' learning [1]. With the reform and deepening of China's teaching system, teachers' evaluation methods and contents are becoming more and more perfect. English teaching quality is constantly changing according to the teaching needs. Teaching quality evaluation system can help teachers understand students' learning situation and obtain students' real reflection information on teaching content, so as to improve teaching methods and teaching content and improve English teaching effect [2]. In addition, schools can analyze and train teachers' teaching according to the results of teaching quality evaluation, help English teachers improve teaching quality and professional quality more scientifically and reasonably, improve teaching management level, and provide new ways for schools to improve teaching quality and development and reform [3, 4].

In the past, the evaluation of English teaching quality was usually directly established by mathematical model, such as analytic hierarchy process, index weighted average method, and fuzzy comprehensive evaluation [5, 6]. These teaching quality evaluation models need a linear relationship between the evaluation index and the influencing factors, but the English teaching quality evaluation belongs to a nonlinear relationship, which cannot reduce the randomness and subjectivity of the influencing factors, so that the final evaluation results and the actual situation show deviation or even distortion [7]. The first problem is that the traditional subject of English teaching quality evaluation is relatively single. In the traditional evaluation system, the evaluation subject is often the expert group, the teacher group, or the student group. The composition of the evaluation subject is single, and it cannot be used to evaluate the quality of English teaching [8, 9]. The second problem is that the indicators of English teaching quality evaluation system are not comprehensive; that is, the content of evaluation indicators of various schools is similar, and the content is relatively simple and more inclined to the theoretical evaluation of teaching, ignoring the characteristics of different disciplines of teaching and making the evaluation content not objective and comprehensive [10, 11]. The third problem is the distortion of the evaluation results of English teaching quality; that is, although the students, as one of the evaluation subjects, feel the most intuitive, profound, and detailed English teaching content, their evaluation objectivity needs to be determined [12]. On the one hand, because of the teacher's strictness, students have resistance emotion, which is too subjective in the evaluation. On the other hand, students' evaluation may mislead teachers, make teachers' requirements for students lower or cater to students' needs too much, and eventually lead to adverse effects on teaching effect [13].

In view of the problems existing in the traditional English teaching quality evaluation method, BP neural network algorithm can give a better solution where neural network algorithm is a kind of network information data processing system with high nonlinear dynamic processing ability. Different from linear relation algorithm, when the variable relationship and distribution form of data are uncertain or when some complex systems cannot express the relationship between input and output data with general relation, BP neural network algorithm cannot express the relationship between input and output data with general relation; neural network can still easily express the highly nonlinear mapping relationship between these data [14]. At the same time, the neural network algorithm can obtain the corresponding experience through the learning of the previous data samples, skip the cumbersome operation of the query and related expression process, and express the data sample law function close to the function that can present the best data state. The characteristics of BP neural network are mainly shown in the following points. The first point is that the nonlinear characteristics of BP neural network can make it infinitely close to any continuous nonlinear function under any given precision condition [15]. The second point is that BP neural network adopts parallel distributed processing method for information storage and processing, which means that BP neural network has strong performance and fast processing speed in information processing, and it shows strong fault tolerance for information [16]. The third point is that the ability of BP neural network to process data can be obtained through learning performance, and it has strong adaptability. It can express different regular data through weight and realize weight Generalization Application [17]. The fourth point is that BP neural network also shows strong data fusion in information processing, which shows that BP neural network can not only use traditional numerical operation skills, but also use artificial intelligence technology to process information quantitatively and qualitatively [18]. The fifth point is that BP neural network is not a single variable system; the number of output and input variables is not fixed, which provides a new general description method for the decoupling problem between subsystems [19]. Therefore, in the evaluation of English teaching quality, the nonlinear characteristics of BP neural network can build the corresponding model in the case of unclear data generation reasons and then through the learning and training of sample data to achieve the desired effect and can effectively reduce the impact of human subjective factors on the final evaluation results, so as to get more comprehensive, reasonable, and scientific results [20, 21].

Although BP neural network has been widely used in many fields and has achieved good results, it still shows some shortcomings in the application process and needs to be improved. Therefore, this paper uses genetic algorithm (GA) to improve the BP neural network algorithm; at the same time, further adaptive mutation optimization is carried out on the GA algorithm, combined with entropy method to screen the optimized GA-BP neural network algorithm data, so as to reduce the error of the optimized GA-BP neural network algorithm and reduce the influence of special individuals and randomness, so as to improve the accuracy and rationality of English teaching quality evaluation system based on GA-BP neural network algorithm.

## 2. Optimize GA-BP Neural Network Algorithm to Build English Teaching Quality Evaluation Model

### 2.1. Construction of English Teaching Quality Evaluation Model Based on 2.1 BP Neural Network Algorithm

BP neural network algorithm is a feedforward artificial neural network based on biological brain neurons, which is a parallel and distributed network structure composed of multiple neurons and can process information [22]. The structure of a single neuron in BP neural network is relatively simple, as shown in Figure 1. At the same time, the function it can achieve is also very simple. However, after different numbers of neurons are connected, its overall performance is not a simple result of one plus one, but a highly complex nonlinear relationship [23].

Each neuron has a single output, but it can be connected with other neurons. It has multiple input paths, and each connection path has a corresponding weight. When the weight value is greater than 0, it means excitation, and when it is less than 0, it means inhibition. As shown in formulas (1)–(3), there is no difference between the two methods.

(1) $$\begin{array}{c} u_{k}=\overset{p}{\underset{j=1}{\sum }}w_{kj}x_{j}, \end{array}$$

(2) $$\begin{array}{c} v_{k}=u_{k}-\theta_{k}, \end{array}$$

(3) $$\begin{array}{c} y_{k}=\varphi \left(v_{k}\right). \end{array}$$

The input signal is expressed as *X*=(*x*_1_, *x*_2_,…,*x*_*p*_)^*T*^, the weight of neuron *k* is expressed as *w*_*k*1_, *w*_*k*2_,…, *w*_*kp*_, the linear combination result is expressed as *u*_*k*_, the threshold value is expressed as *θ*_*k*_, the excitation function is expressed as *φ*(*v*_*k*_), and the output of neuron is expressed as *y*_*k*_. There are threshold function, piecewise linear function, and *S*-type function in incentive function. According to the requirements of this paper and the performance of different incentive functions, this paper selects *S*-type function as incentive function, as shown in the following formula:

(4) $$\begin{array}{c} \varphi \left(v\right)=\frac{1}{1+\exp\left(-v\right)}. \end{array}$$

BP neural network can be divided into three layers, namely, input layer, hidden layer, and output layer, and each layer contains a number of neurons that do not have any connection with each other. Neurons of each layer are only connected with neurons of adjacent levels, and the information transmission is unidirectional without feedback [24]. The topological structure of BP neural network is shown in Figure 2.

Before the sample training of BP neural network, it is necessary to initialize the network and the corresponding learning parameters and determine the fixed parameters. BP neural network training samples mainly include input vector *X*=[*x*_1_, *x*_2_,…,*x*_*n*1_]^*T*^ and expected output vector *T*=[*t*_1_, *t*_2_,…,*t*_*N*3_]^*T*^. The output formula of the nodes in the hidden layer is shown as follows:

(5) $$\begin{array}{c} y_{h}^{k}=f\left(\overset{N1}{\underset{i=1}{\sum }}w_{ih}\cdot x_{i}^{k}+\theta_{h}\right), \end{array}$$

where *k* is the number of corresponding samples and *k*=1,2,…, *N*, *θ*_*h*_ is the threshold, and *f* is the transfer function. The node output formula of the output layer is shown as follows:

(6) $$\begin{array}{c} o_{s}^{k}=g\left(\overset{N2}{\underset{h=1}{\sum }}w_{hs}\cdot y_{h}^{k}+\theta_{s}\right), \end{array}$$

where *k* is the *k*-th sample and *k*=1,2,…, *N*, *θ*_*s*_ is the threshold, and *g* is the transfer function.

The error function of BP neural network is shown as follows:

(7) $$\begin{array}{c} E_{s}=\frac{1}{2}\overset{N3}{\underset{S=1}{\sum }}\left(T_{s}^{k}-O_{S}^{K}\right). \end{array}$$

The error function of global sum of squares error *E* is given by

(8) $$\begin{array}{c} E=\frac{1}{2}\overset{N}{\underset{k=1}{\sum }}\overset{N3}{\underset{S=1}{\sum }}\left(T_{s}^{k}-O_{S}^{K}\right). \end{array}$$

When there is a gap between the output value of the output layer and the expected value, it is necessary to calculate the correction error, as follows:

(9) $$\begin{array}{c} d_{s}^{k}=\left(t_{s}^{k}-o_{s}^{k}\right)o_{s}^{k}\left(1-o_{s}^{k}\right), \end{array}$$

where *s*=(1,2,…, *N*_3_). Thus, the correction error of the hidden layer can be obtained as follows:

(10) $$\begin{array}{c} e_{h}^{k}=\left[\overset{n3}{\underset{s=1}{\sum }}d_{s}^{k}w_{hs}^{k}\right]y_{h}^{k}\left(1-y_{h}^{k}\right). \end{array}$$

The weight and threshold of BP neural network algorithm are calculated by gradient descent algorithm, and its iteration period is shown as follows:

(11) $$\begin{array}{c} w^{k+1}=w^{k}+\Delta w=w^{k}-\eta^{k}\frac{\partial e^{k}}{\partial w^{k}}, \end{array}$$

where *w*^*k*^ is the weight vector or threshold vector of *k* times, *η*^*k*^ is the learning rate of corresponding times, and ∂*e*^*k*^/∂*w*^*k*^ is the error gradient. It can be seen that the BP neural network algorithm has a flat error area; that is, the error is still in a slow decline state when the weight is maximum, which greatly increases the number of trainings and affects the convergence speed. In addition, the BP neural network algorithm has a greater probability of falling into the local minimum problem, so that there is a certain gap between the training convergence result and the expected error. Because of falling into the concave point of the error surface, the activation function of neural network is *s* function. Both ends of this function are flat, and the algorithm runs very slowly. As long as it is a random search algorithm, this will happen, but the possibility is different. It can use the advance search with strong global optimization ability and then use the algorithm with strong local search ability to continue the search.

### 2.2. Optimization of GA-BP Algorithm English Teaching Quality Evaluation Model

According to the above problems of BP neural network algorithm, this paper uses GA algorithm to optimize BP neural network algorithm. When the structure of BP neural network is *x* − *y* − 1, the number of weights is(*x∗y*+*y*). The number of thresholds is(*y*+1). Then the total length is shown as follows:

(12) $$\begin{array}{c} \text{LEN}=\left(x*y+y\right)+\left(y+1\right). \end{array}$$

Then, the sum of the absolute error of the BP neural network algorithm after training is taken as the individual fitness value, as shown in the following formula:

(13) $$\begin{array}{c} F=k\overset{n}{\underset{i=1}{\sum }}\left(y_{i}-o_{i}\right), \end{array}$$

where *n* indicates the number of output nodes, *y*_*i*_ represents the ideal output, *o*_*i*_ represents the predicted output, and *k* represents the coefficient. The selection, crossover, and mutation of GA algorithm are shown in formulas (14)–(16):

(14) $$\begin{array}{c} \text{pselect}=\frac{f_{i}}{\sum_{j=1}^{N}f_{i}}. \end{array}$$

Among them, pselect represents the selection probability of individuals in a population, *f*=*k*/*F*_*i*_ and *F*_*i*_ represents the individual fitness value, *k* is the coefficient, and *N* represents the number of individuals in a population.

(15) $$\begin{array}{c} a_{mj}=a_{mj}\left(1-b\right)+a_{nj}b,\\ a_{nj}=a_{nj}\left(1-b\right)+a_{mj}b. \end{array}$$

In the above formula, the coding method is real number coding; that is, chromosomes *a*_*m*_ and *a*_*n*_ are mutated at *j* position, *b* is a random number, and the range is [0, 1].

(16) $$\begin{array}{c} \left\{\begin{array}{cc} a_{ij}=a_{ij}+\left(a_{ij}-a_{\max}\right)*f\left(\text{ga}\right), & \text{rand}>0.5,\\ a_{ij}=a_{ij}+\left(a_{\min}-a_{ij}\right)*f\left(\text{ga}\right), & \text{rand}<0.5, \end{array}\right) \end{array}$$

where *a*_*ij*_ is the *i* gene of the *j*-th individual, *a*_max_ is the upper limit of *a*_*ij*_, *a*_min_ is the lower limit of *a*_*ij*_, *f*(ga)=*r*(1 − ga/ga_index)^2^, and *r* is a random number, ga is the current number of iterations, ga_index is the maximum number of iterations, and rand is a random number with the range of [0, 1].

In the GA algorithm, the adaptability of the population has a great influence on its search for the global optimal solution. When the fitness is good, that is, when the global optimal solution is nearest, the GA algorithm can be further optimized by adaptive mutation. As shown in formula (17), the adaptive mutation probability calculation formula is as follows:

(17) $$\begin{array}{c} Q=\frac{Q_{1}+Q_{2}}{2}=\frac{\left\{Q_{0}-\left(Q_{0}-Q_{\min}\right)\times \left(\text{ga}/\text{ga\_index}\right)+Q_{0}\times \left(\bar{F}/\max_{X_{k}\in \Omega }F\left(X_{k}\right)\right)\right\}}{2}. \end{array}$$

Among them, ga represents the current number of iterations, ga_index represents the maximum number of iterations, *Q*_min_ represents the minimum value in the variation range, $\bar{F}$ represents the average fitness value of the population, and max_*X*_*k*_∈Ω_*F*(*X*_*k*_) represents the maximum fitness value of the population.

The index information of the evaluation system of English teaching quality is relatively large, and there are many influencing factors in the comprehensive evaluation. If the data is directly input into the GA-BP neural network algorithm, some special data will increase the error of the algorithm and slow down the convergence speed, so the data should be processed before the training and learning. In this paper, the entropy method is used to process the data, that is, to avoid the randomness and subjectivity of the data on the basis of the given index weight of the data, and then the GA-BP neural network algorithm is used for learning and training, as shown in the following formula:

(18) $$\begin{array}{c} x{}^{\prime }{}_{pq}=\frac{x_{pq}-\bar{x}}{s_{q}} \end{array}$$

Among them, *x*_*pq*_ represents the score of the *p* sample on the *q*-index, *x*′_*pq*_ represents the standardized value, $\bar{x}$ represents the average value, and *s*_*q*_ represents the standard deviation. The average value shift after standardization is shown in the following formula:

(19) $$\begin{array}{c} Z_{pq}=x{}^{\prime }{}_{pq}+A, \end{array}$$

where *A* is the translation length.

The proportion of the *p* sample in *q* index is shown in the following formula:

(20) $$\begin{array}{c} P_{pq}=\frac{Z_{pq}}{\sum_{i=1}^{n}Z_{pq}}. \end{array}$$

The entropy value of the *q* index is shown as follows:

(21) $$\begin{array}{c} E_{j}=-k\overset{n}{\underset{i=1}{\sum }}P_{pq}\ln\left(P_{pq}\right). \end{array}$$

The difference value of the *q* index is shown as follows:

(22) $$\begin{array}{c} G_{j}=1-E_{j}. \end{array}$$

After normalizing the difference value, the weight of the *q* indicator is shown as follows:

(23) $$\begin{array}{c} w_{j}=\frac{G_{j}}{\sum_{j=1}^{m}G_{j}}. \end{array}$$

Then the teaching quality of the *p* sample is shown as follows:

(24) $$\begin{array}{c} H_{i}=\overset{m}{\underset{j=1}{\sum }}w_{j}P_{pq}. \end{array}$$

Figure 3 shows the flowchart of English teaching quality evaluation based on optimized GA-BP neural network algorithm.

### 2.3. Construction of Structural Model and Evaluation Index of English Teaching Quality Evaluation System

The evaluation of English teaching quality involves English teaching leaders, namely, teachers, English teaching audiences, namely, students, English teaching experts, and other English teachers. Therefore, the objects of English teaching quality evaluation need to be composed of different groups. As shown in Figure 4, it is the structural model of English teaching quality evaluation system.

It can be seen from the figure that the system is divided into two levels. The input information starts from the level 2 indicators, and the output of each level 2 indicator is the corresponding level 1 indicator information. The final result of English teaching quality is divided into excellent, good, general, pass, and fail. The output value range of GA-BP neural network corresponding to each level is shown in Table 1.

There are many influencing factors in the process of English teaching and learning, such as English teaching methods, teaching content difficulty level, teachers' professional quality, students' English foundation, students' interest in English learning, and so on. Therefore, according to the characteristics of English teaching and the needs of students, the evaluation index of English teaching quality is constructed, as shown in Figure 5.

## 3. Simulation Results of English Teaching Quality Evaluation System Based on Optimized GA-BP Algorithm

### 3.1. Algorithm System Training Results

According to Figure 5, we can see that there are 17 secondary indexes of English teaching quality evaluation index, then the corresponding optimized GA-BP neural network algorithm has 17 input layer nodes, 1 output layer node, and 5 hidden layer nodes, the maximum number of iterations is 120 and the accuracy is 10–8, the real coding length of GA algorithm is 80, the initial scale is 22, and the cross probability is 0.7. As shown in Figures 6 and 7, the mean square errors of GA-BP neural network and optimized GA-BP neural network are shown, respectively.

It can be seen from Figure 6 that the mean square error of GA-BP neural network algorithm decreased greatly in the first five iterations. From the fifth to the twenty-seventh iterations, the mean square error of GA-BP neural network algorithm decreased slightly, gradually tended to a gentle decline state, and reached convergence in the thirty-fifth iteration. In the first five iterations, the mean square error of the optimized GA-BP neural network algorithm decreases rapidly and then decreases slowly until the 20th iteration and reaches the convergence state in the 25th iteration. This shows that the optimized GA-BP neural network algorithm has a faster mean square error reduction rate than GA-BP neural network algorithm, improves the convergence speed of the algorithm, and can achieve the convergence effect in fewer iterations.

As shown in Figures 8 and 9, the fitness diagrams of GA-BP neural network algorithm and optimized GA-BP neural network algorithm are shown. It can be seen from the figure that the GA-BP neural network algorithm has a faster convergence speed in the first 40 iterations and gradually tends to be flat from 40 to 50 iterations. After 50 iterations, it is stable, and the final fitness value is 0.83. The convergence speed of the optimized GA-BP neural network algorithm is faster, reaching a stable state in the 20th iteration, and the fitness value reaches 1.43. This shows that the optimized GA-BP neural network algorithm model has faster convergence speed than GA-BP neural network algorithm model under the condition of the same genetic times, can reach a stable state in a shorter time, and has higher fitness value; that is, the optimized GA-BP neural network algorithm model has higher adaptability.

### 3.2. Experimental Results of English Teaching Quality Evaluation System Based on Optimized GA-BP Neural Network Algorithm

Genetic algorithm optimizes BP, including three parts: neural network structure determination, genetic algorithm optimization, and BP neural network prediction. Among them, genetic algorithm is used to optimize the initial weight and threshold of BP neural network, so that the optimized BP neural network can better predict the function output. The purpose of optimizing BP neural network by genetic algorithm is to obtain better network initial weight and threshold through genetic algorithm. Its basic idea is to use the initial weight and threshold of individual representative network and the prediction error of BP neural network initialized by individual value as the fitness value of the individual and find the optimal individual through selection, crossover, and mutation operations, that is, the optimal initial weight of BP neural network.

In order to effectively verify the effect of the English teaching quality evaluation system based on the optimized GA-BP neural network algorithm, this paper selects 15 sample data for learning and training and another 8 groups of data for simulation experiments. As shown in Figure 10, it is the result of GA-BP neural network algorithm and optimized GA-BP neural network algorithm after learning and training 15 groups of sample data.

It can be seen from the figure that the prediction results of GA-BP neural network algorithm after sample learning and training are similar to the ideal results as a whole, but the error of individual prediction results is large; in particular the data error of samples 6 to 10 is the largest, which indicates that GA-BP neural network algorithm is greatly affected by individual factors. The prediction result of optimized GA-BP neural network algorithm is closer to the ideal result, both the overall sample error and individual sample error are relatively small, and it is more stable than GA-BP neural network algorithm. Therefore, the evaluation system model of English teaching quality based on optimized GA-BP neural network has higher value in application, and the evaluation of English teaching quality is more scientific.

Figure 11 shows the performance comparison table of different English teaching quality evaluation models. From the data in the table, it can be seen that, in the BP neural network algorithm, GA-BP neural network algorithm, and optimized GA-BP neural network algorithm, the average evaluation accuracy of optimized GA-BP neural network algorithm is the highest, and it is 15.29% and 7.37% higher than BP neural network algorithm and GA-BP neural network algorithm, respectively. This shows that the optimized GA-BP neural network has better evaluation performance.

Figure 12 shows the simulation experiment results of eight groups of data by the English teaching quality evaluation system based on the optimized GA-BP neural network algorithm. It can be seen from the figure that the error of the test sample is very close to the training error, and the prediction accuracy of both the training and the test results is within the allowable range, and there is no individual error increase. This shows that the English teaching quality evaluation system based on optimized GA-BP neural network algorithm is reasonable, scientific, and feasible.

## 4. Conclusion

With the continuous improvement of China's economic level and international status, people have more and more opportunities to choose to communicate in their study, work and life, study, tourism, etc. The importance of English is becoming more and more prominent. As one of the important contents of basic education in China, English teaching quality level and teaching content are related to the ultimate goal of English teaching, so the construction of English teaching quality evaluation system has been widely concerned. The traditional English teaching quality evaluation system mainly analyzes and evaluates the data by constructing linear mathematical model, but this way cannot reduce the influence of subjective factors in the data to the minimum and cannot comprehensively analyze and consider the nonlinear factors, which makes the evaluation results of English teaching quality not comprehensive and does not conform to the characteristics of English teaching. Even the result of English teaching quality evaluation is distorted. Therefore, in view of the above problems, this paper studies the English teaching quality evaluation system based on the optimized GA-BP neural network algorithm. The nonlinear characteristics of BP neural network can well reflect the nonlinear relationship between the evaluation index and the result of English teaching quality and reduce the randomness and subjectivity of influencing factors. At the same time, in order to solve and improve the convergence speed and global optimal solution of BP neural network, this paper optimizes BP neural network by GA algorithm. In addition, combined with GA adaptive mutation optimization and entropy method, the prediction effect of GA-BP neural network is further improved to achieve the purpose of optimization. The experimental results show that, compared with GA-BP neural network algorithm, the optimized GA-BP neural network has better performance in both convergence speed and mean square error. At the same time, under the condition of the same number of iterations, the optimized GA-BP neural network algorithm fitness value can achieve stable effect faster and has higher fitness value; that is, it has better adaptive ability. After training, the sample test results show that the prediction value of the optimized GA-BP neural network algorithm is closer to the ideal value, with higher accuracy and better stability. It shows greater application value in the English teaching quality evaluation system, and the evaluation results are more scientific and reasonable. However, the probability of BP neural network algorithm falling into the local minimum problem is large, so there is a certain gap between the training convergence result and the expected error, a concave point that falls into the error surface. The activation function of neural network is *s* function. Both ends of the function are flat, and the algorithm runs very slowly. As long as it is a random search algorithm, this will happen, but the possibility is different. Use the advanced search with strong global optimization ability and then continue the search with the algorithm with strong local search ability. This needs to be improved in future research.

## Figures and Tables

**Figure 1:** Simple model of the neuron.

**Figure 2:** BP neural network topology.

**Figure 3:** English teaching quality evaluation flowchart based on the optimized GA-BP neural network algorithm.

**Figure 4:** The structural model of English teaching quality evaluation system.

**Figure 5:** The evaluation index of English teaching quality.

**Figure 6:** GA-BPNN mean square error.

**Figure 7:** The mean square error of GA-BPNN was optimized.

**Figure 8:** The fitness of GA-BPNN.

**Figure 9:** The fitness of GA-BPNN was optimized.

**Figure 10:** Comparison of prediction results between GA-BP neural network algorithm and optimized GA-BP neural network algorithm.

**Figure 11:** Performance comparison table of different English teaching quality evaluation models.

**Figure 12:** The simulation results of English teaching quality evaluation system based on the optimized GA-BP neural network algorithm.

**Table 1:** The corresponding table of grading standards and GA-BPNN output values.

Level	GA-BPNN output values
Excellent	1.00–0.90
Good	0.89–0.80
Fair	0.79–0.70
Pass	0.69–0.60
Fail	<0.59

## Data Availability

The data used to support the findings of this study are available from the corresponding author upon request.
